The article "Explainable AI in Diagnosing and Anticipating Leukemia Using Transfer Learning Method" was retracted in 2023. Reasons: signs of a paper mill; compromised peer review; unreliable results or conclusions.

# Explainable AI in Diagnosing and Anticipating Leukemia Using Transfer Learning Method

**DOI:** 10.1155/2022/5140148

**Published:** 2022-04-27

**Authors:** Wahidul Hasan Abir, Md. Fahim Uddin, Faria Rahman Khanam, Tahia Tazin, Mohammad Monirujjaman Khan, Mehedi Masud, Sultan Aljahdali

**Affiliations:** ^1^Department of Electrical and Computer Engineering, North South University, Bashundhara, Dhaka-1229, Bangladesh; ^2^Department of Computer Science, College of Computers and Information Technology, Taif University, P. O. Box 11099, Taif 21944, Saudi Arabia

## Abstract

White blood cells (WBCs) are blood cells that fight infections and diseases as a part of the immune system. They are also known as “defender cells.” But the imbalance in the number of WBCs in the blood can be hazardous. Leukemia is the most common blood cancer caused by an overabundance of WBCs in the immune system. Acute lymphocytic leukemia (ALL) usually occurs when the bone marrow creates many immature WBCs that destroy healthy cells. People of all ages, including children and adolescents, can be affected by ALL. The rapid proliferation of atypical lymphocyte cells can cause a reduction in new blood cells and increase the chances of death in patients. Therefore, early and precise cancer detection can help with better therapy and a higher survival probability in the case of leukemia. However, diagnosing ALL is time-consuming and complicated, and manual analysis is expensive, with subjective and error-prone outcomes. Thus, detecting normal and malignant cells reliably and accurately is crucial. For this reason, automatic detection using computer-aided diagnostic models can help doctors effectively detect early leukemia. The entire approach may be automated using image processing techniques, reducing physicians' workload and increasing diagnosis accuracy. The impact of deep learning (DL) on medical research has recently proven quite beneficial, offering new avenues and possibilities in the healthcare domain for diagnostic techniques. However, to make that happen soon in DL, the entire community must overcome the explainability limit. Because of the black box operation's shortcomings in artificial intelligence (AI) models' decisions, there is a lack of liability and trust in the outcomes. But explainable artificial intelligence (XAI) can solve this problem by interpreting the predictions of AI systems. This study emphasizes leukemia, specifically ALL. The proposed strategy recognizes acute lymphoblastic leukemia as an automated procedure that applies different transfer learning models to classify ALL. Hence, using local interpretable model-agnostic explanations (LIME) to assure validity and reliability, this method also explains the cause of a specific classification. The proposed method achieved 98.38% accuracy with the InceptionV3 model. Experimental results were found between different transfer learning methods, including ResNet101V2, VGG19, and InceptionResNetV2, later verified with the LIME algorithm for XAI, where the proposed method performed the best. The obtained results and their reliability demonstrate that it can be preferred in identifying ALL, which will assist medical examiners.

## 1. Introduction

Blood supplies essential substances to the entire human body. Erythrocytes (red blood cells), leukocytes (white blood cells), and thrombocytes (platelets) are the three main components of blood cells in the human body. In the human body, red blood cells (RBCs) ensure oxygen transportation to different parts of the body, and in the case of injury, platelets help with blood clotting. White blood cells (WBCs) fight germs and prevent human infections. WBCs make up only 1% of blood volume, but slight changes are significant because the human immune system depends on WBCs. Any fluctuation in the number of leukocytes (WBCs) in the blood indicates a problem. Having an abnormally high number of WBC in our bodies can be detrimental and contribute to disease. Among them, leukemia is one of the most common diseases related to WBC count [1]. Leukemia is a prevalent and deadly disease. Leukemia is a cancer of leukocytes (WBCs) that affects the blood-forming cells. Many teenagers and children are at risk of developing leukemia. According to a 2012 study [2], around 352,000 people and children worldwide get leukemia, which begins inside the bone marrow and is identified by an unexpected growth in the number of white blood cells. These defective blood cells put the immune system at risk, which affects the blood and bone marrow. Furthermore, these malignant WBCs can enter the bloodstream, and these cancerous cells can spread to multiple organs and harm the entire body via infected blood cells, which can be threatening if not diagnosed early or if therapy is delayed [3].

Leukemia is classified primarily based on whether it is increasing rapidly (acute) or slowly (chronic). Each of these types can be fatal if not detected or if therapy is delayed. Chronic leukemia usually takes a long time to develop. In contrast, the average survival time for acute leukemia patients without specific treatment is only three months. Acute lymphocytic leukemia is the most common among children, accounting for 25% of all childhood cancers [4]. ALL can lead a patient to death. If it is detected early on, it is generally treatable, and the patient's chances of survival increase. That is why early detection of immature cell formations is necessary to increase the patients' survival rate. Early and accurate diagnosis could help patients save money on therapy and increase their chances of remission. The limitations of diagnosing leukemia patients by humans are time-consuming and can become error-prone. An inaccurate diagnosis can threaten a patient's health. And in addition to making treatment more difficult, it raises treatment expenses. Hence, developing automated, low-cost systems that can accurately identify healthy and abnormal blood smear images is crucial. Many assisting systems have been proposed to aid physicians in achieving high diagnosis accuracy. Physicians can diagnose a disease based on a specific dataset that includes signs, symptoms, medical images, and exams.

Many researchers have proposed many strategies and algorithms for recognizing, segmenting, and classifying ALL. The success of classification is dependent on the success of feature extraction, which is dependent on the success of segmentation. Hence, high classification accuracy requires the execution of all procedures. Deep learning has recently achieved remarkable progress in computer vision, image processing, and recognition. It has become a promising choice for medical image analysis [5]. Among them, a considerable amount of work has been focused on leukemia diagnosis. Some researchers use the CNN method to diagnose leukemia. CNN is the most extensively used method for image recognition. It has high self-learning, adaptability, and generalization abilities. Traditional image recognition methods need feature extraction and classification, whereas CNN [6] requires only the image data as an input to complete the image classification with the network's self-learning ability. For example, Nayaki et al. [7] demonstrated a DL system based on image processing and CNN methods to detect defective blood cells in microscopic blood images and achieved an accuracy rate of 80.4%. Kasani et al. presented [8] a study to classify leukemic B-lymphoblast to develop an aggregated DL model. They created a trustworthy and accurate deep learner that can correctly diagnose ALL with a 96.58% classification accuracy using a small dataset size. Hegde et al. [9] have compared traditional image processing approaches and DL methods in the task of classifying WBCs. They achieved a significant performance increase over traditional methods using neural network architecture. Macawile et al. [10] proposed a WBC classification and counting method using pretrained CNN. They used modified AlexNet, GoogLeNet, and ResNet-101 in tandem to obtain classification results. Sharma et al. [11] applied a custom CNN architecture for WBC classification; the proposed network consists of 2D convolutions and MaxPooling layers with ReLU activations. This architecture achieved high accuracy scores for binary and multiclass classification settings. Genovese et al. [12] have introduced the first method for ALL detection based on histopathological transfer learning. On a histopathology database, CNN is trained before being fine-tuned on the ALL database to recognize lymphoblast tissue types with an accuracy rate of 88.69%. Safuan et al. [13] classified the WBC types to identify ALL with CNN, where pretrained models of DL like AlexNet, GoogLeNet, and VGG-16 are differentiated from each other to find the model that can classify better with a classification accuracy rate of 96.15%. Shafique and Tehsin [14] compared the different methods for the early detection of ALL. The various stages in the diagnosis procedure are comparatively analyzed in their study. They also discuss the advantages and disadvantages of each method. Jiang et al. have proposed [15] the ViT-CNN ensemble model to help diagnose ALL by classifying cancerous and normal cells. The ViT-CNN ensemble model extracts features from cell pictures in two alternative ways to improve classification, resulting in a very accurate detection method with 99.03% accuracy. Aftab et al. have proposed [16] a methodology for detecting leukemia using the Apache Spark BigDL library and CNN architecture for GoogLeNet deep transfer learning. They used microscopic images of human blood cells and reached a 96.42% accuracy rate. However, the lack of explainability of neural networks limits the wide-scale adoption of DL in healthcare applications where explaining the fundamental logic is vital for decision-making. DL models are often considered “black boxes model”, which are tough to decipher. There is no clear dividing line when a model becomes a black box. Even when the model's structure and weights are obvious, complex models like machine learning (ML) or DL, with hundreds or even millions of parameters, are considered “black boxes” because their behavior is difficult to explain [17]. Among them, the neural networks used in DL are the most difficult to comprehend. If AI cannot explain itself in the healthcare domain, the risk of making a wrong decision may outweigh the benefits of precision, speed, and decision-making efficacy. As a result, its scope and utility would be severely limited. That is why XAI [18] can help better understand and explain DL and neural networks. The adoption of XAI techniques is justified by the desire to promote transparency, result tracking, and model improvement. For example, Pawar et al. discussed [19] XAI as a technique for AI-based systems to analyze and diagnose health data to provide accountability, transparency, result tracking, and model improvement in the healthcare domain. Besides, Arrieta et al. proposed an analysis of recent contributions to different ML models' explainability. These models focused on explaining various DL methodologies [20]. So, these intelligent healthcare systems can then be utilized to diagnose leukemia and choose the best treatment option. XAI can explain both the diagnosis result and the radix of the prediction. One of the first two major initiatives in the history of XAI was LIME [21]. A DL model's predictions are made with the help of LIME, a tool that can find features in an image or text. It is not limited to a single model. It can be used with a wide range of ML and DL algorithms. LIME aims to figure out what the model's most essential features are or what the primary components that drive any particular choice are. This strategy can clarify whether the model's predictions are based on a single phrase in a document or a characteristic in an image. Deep neural network construction and training are time-consuming and very complex processes. So, instead of creating a deep neural network from scratch, the concept of transfer learning can be applied, where a deep network that has successfully solved one problem is customized to solve another.

The proposed approach in this paper aims to implement and compare different transfer learning models of TensorFlow in classifying acute lymphocytic leukemia (ALL) which will help doctors detect ALL cells in patients to save human lives. By comparing different transfer learning models, future research on ALL classification will get a head start in choosing transfer learning models. Also, this method manages to explain which part of the image from the dataset caused the model to make a specific classification using LIME to assure the model's validity and reliability. As deep learning in terms of medical classification is getting more popular; it is very important to know the cause of a prediction so that the doctor can easily verify the result. This procedure will make ALL classification easier, more accurate, and more reliable. The main motivation of this paper is to help medical experts detect ALL, not only with high accuracy but also with proper explanation by using XAI. As XAI directly points at the affected cell portion, this study informs doctors about the sample cell to make an accurate conclusion while trusting the deep learning model. The study further helps future researchers in choosing deep learning models for medical complications by comparing different models on ALL detection.

The main objective of the proposed method is to compare different transfer learning methods with high accuracy and an F1 score, which can identify ALL. The proposed method uses stratified KFold and XAI to showcase the image concentration of sample cells, which is novel in classifying leukemia with high precision. The use of XAI makes the proposed method very reliable for medical examiners. There is no research yet on ALL that has both high accuracy and uses XAI even though the dataset is imbalanced. By involving the stratified KFold method in ALL, this study showcases a superior way to train models in medical care. Also, the proposed method handles imbalanced datasets smoothly in a very modern way. It reduces costs and saves time by automating the process. Also, comparison between different transfer learning methods helps future researchers choose suitable leukemia research methods, which contributes to paving the way for further improvement.

The remaining contents of the paper are arranged as follows: Section 2 proposes the method and materials. This section gives a gist of the system model and the whole system. Then, the results and analysis are described in Section 3. Lastly, in Section 4, the paper ends with the conclusion.

## 2. Materials and Methodology

### 2.1. Dataset Description

The dataset used for leukemia cancer identification was obtained from the open-source website Kaggle [22] to train and test the model, which was used for the ALL challenge of ISBI 2019 [23].

These cells were segmented from microscopic images and are indicative of real-world photos since they contain staining noise and illumination flaws, but these faults were mostly addressed after acquisition. This is because morphological similarities make it difficult to distinguish young leukemic eruptions from normal cells under a microscope. An expert oncologist annotated the ground truth labels. There are 15,114 photos in all from 118 patients, divided into two classes: normal cell and leukemia blast cell. The photos in the dataset are 450px *x* 450px and in bmp format. In Figure 1, there are sample images from two classes.

### 2.2. Proposed Framework

The focus of this method is to detect ALL using transfer learning and later validate the model using XAI. Firstly, the leukemia images were collected from the CNMC website. As the dataset was imbalanced with the more ALL class, the class weight method was used to balance the weights of the two classes in preprocessing. The class weight function was followed because it is an optional dictionary mapping class, mostly used for the loss function during training. It is one of the most efficient techniques for dealing with an imbalanced dataset. From Sklearn, a compute_class_weight function with parameters of “balanced” was used.

(1) $$\begin{array}{c} \text{Class}\_\text{weight}=\frac{n\_\text{samples}}{\left(n\_\text{classes }*np.\text{bincount}\left(y\right)\right)}. \end{array}$$

For the used dataset, the class weight of normal cells was 1.57288, and the class weight of acute lymphocytic leukemia (ALL) cells was 0.73301.

Then, different pretrained models, namely InceptionV3, ResNet101V2, VGG19, and InceptionResNetV2, were used to train the model. For further validation and explanation of the model, the LIME algorithm was used, where the model indicates the focus point in a sample cell.

Figure 2 shows the overall block diagram of the framework followed for this research. After collecting the dataset, the dataset went through preprocessing to ensure proper feature selection. Image augmentation was performed as feature engineering to make the model more robust in detecting unseen samples. Later, using stratified Kfold, the dataset was split into 3 folds. The model was built with specific hyperparameters to be trained. Finally, it was tested on unseen sample cells, and its reliability was verified using XAI.

### 2.3. Data Preprocessing

All the images were reduced to 299px *x* 299px, because the InceptionV3 input shape must be (299, 299, 3) and a standard batch size of 32 is used while training. For RGB images, the channel size should be 3. Up to this point, the images were not binarily labeled, so ALL cells and normal cells were labeled 1 and 0 correspondingly. Labeling the dataset makes it easy to understand, and all the data points are simplified to a standard value.

### 2.4. Data Splitting

It can be difficult to assess a DL model. Typically, the dataset is usually partitioned into testing and training sets. The model is trained using a training set, and model testing is performed using the testing set. Then, the correctness of the model is determined by evaluating its performance using an error metric. On the other hand, in a traditional method, the accuracy gained for one test set can be substantially different from another one. K-fold cross-validation [24] offers a solution to this challenge. It separates the data into folds to ensure that each fold is used as a testing set.

### 2.5. Data Augmentation

The proposed method uses TensorFlow data augmentation functions such as random flip (up_down and left_right). While training an image, it is important to use augmentation so that the model can identify a wide range of samples in real-life scenarios. The functions random_flip_up_down() and random_flip_left_right() randomly flip images vertically and horizontally, so that this model, even if a leukemia-affected cell does not fit the training dataset, can still make a correct prediction in practice. A transpose is performed based on the spatial relationship of one image.tf.random.uniform() taking the datatype as float32, and if the spatial value is greater than 0.75, it will perform a transpose. Also, depending on pixel size, saturation, contrast, brightness, and contrast are set. Some sample images may be brighter or more saturated than the training images in the test set. So it is highly beneficial to perform this augmentation of data. For the better focus of the model in the cell, some images underwent cropping functions for better effectiveness, but all images were later resized and reshaped to fit the model. The images were in bitmap image file (bmp) format, and they had to be decoded and converted to the tensor format. A tensor is a multidimensional array. Tensors can represent an image or video as an array [25]. This helps the model read the image easily. Finally, cancel the data duplication and sorting to ensure that the training phase is completely unbiased. If the model is trained using the same image multiple times, the model might be biased to predict test examples according to the repeated data image. Images in all the batches were first converted to a NumPy array along with their labels. The augmentation batch size is the same as the training batch size. Finally, the images were plotted using the Matplotlib library to verify the process after augmentation.  Figure 3 shows the output of dataset images after the augmentation process.

### 2.6. Convolutional Neural Network (CNN)

A convolutional neural network (CNN) is a part of a DL method that takes an image sample as input and assigns priority to different neural features in the sample image, distinguishing between distinct elements. The quantity of preprocessing required by CNN is much smaller than that required by other classification algorithms. While other basic techniques need hand-engineered filters, CNN can acquire these features appropriately [26].

Using CNNs has been very successful in the case of image classification. CNN's strength is its ability to automatically extract high-level information. First, the network architecture needs to be designed before training a CNN for image classification. This task entails determining the network's layer types, numbers, and order. The suggested network seeks to identify features to be utilized for differentiating classes with a set of 2D images and their accompanying class labels. CNN learns by using two repeated and alternated passes, called the “feedforward and backward pass” method. The feedforward pass accomplishes two significant tasks. The primary task is to extract features using many convolutional feature extraction (CFE) layers [27]. For this reason, images are routed serially through many CFE layers. A CFE layer comprises three sublayers: a convolutional layer, a nonlinear transformation layer, and a pooling layer. Each CFE layer creates higher-level features by using features from the previous layer. Extracting advanced information from an image requires frequent repetition of this method. In the second task of the feedforward pass, the fully connected layers use these features to classify the sample image. These have a few errors. The feedforward pass propagates backward previous errors in a backward pass for altering the weights in the convolutional sublayers and allows the extraction of more information concerning the classification problem [28].

InceptionV3 is an extended version of the well-known GoogLeNet, which has shown high classification performance in various biomedical applications using transfer learning. Inception-v3 created an inception model that combines many convolutional filters of various sizes into a single new filter, similar to GoogLeNet. Due to this architecture, the number of training parameters is reduced. Hence, the computational complexity is reduced. The basic architecture [29] of InceptionV3 is demonstrated in Figure 4.

### 2.7. Transfer Learning

A range of applications use deep CNNs because they can learn rich visual representations. However, for medical image-related problems, this needs a huge amount of data to complete the feature extraction for medical image-related problems. The dataset used for leukemia classification is insufficient to achieve good precision, resulting in overfitting the model. To overcome this problem, a transfer learning technique is used in this paper to overcome this problem. Even if the dataset is limited, transfer learning can improve model learning performance by solving the problem of insufficient samples. Transfer learning is a very effective but simple method to improve a network by transferring parameters from one domain (the target domain) to another [30].  Figure 5 shows the working process of conventional ML and transfer learning. In conventional ML, the model is trained from scratch, so the model requires more data to achieve a high score in performance matrices. But on the other hand, in the transfer learning technique, the model already has knowledge from the source task, so it requires very little data for the target task to get high scores in performance matrices.

Adjusting the weight of data in the source domain is essential for usage in the target domain in a discriminatory manner. Transfer learning can outperform the scratch network since the pretrained model already has a lot of basic information. The transfer learning method learns from the transferred domain about both low-end and mid-level properties. A modest amount of data from the new domain is required to achieve better outcomes, which is desirable for this work [31].

The training process for the model was done in batches, with a set batch size of 32. Training in batches allows for computational speedup. Without splitting into batches, the DL algorithm has to store all the error values from 15,114 photos of the dataset in memory. Before training, all the batch images were converted into NumPy arrays. A transfer learning technique is applied in this research as it helps to get better accuracy using fewer data points. In training, some well-known pretrained models have been used. ML models frequently fail to generalize appropriately when applied to data that have not been trained on. It occasionally fails miserably, and at other times it performs only marginally better than abysmal. A resampling technique called cross-validation ensures that the model will perform well on unknown data. This resampling procedure divides the entire dataset into *k* sets of about similar sizes. The model has been trained using the remaining k-1 sets, with the first set serving as the test set. The test error rate is computed after fitting the model to the test data; the test error rate is computed. The second iteration uses the second set as a test set, whereas the remaining k-1 sets are utilized for training the data and determining the error. This method is repeated for all *k* sets. Stratified k-fold CV is used mostly in the event of classification difficulties, including class imbalance. Each training and validation fold ensures that the relative class proportion is nearly maintained. In circumstances where there is a significant class division, it becomes critical. Stratified K-fold cross-validation takes less time to compute and has a lower variance than traditional K-fold cross-validation. Furthermore, because more data points are used for invalidation, the MSE (mean square error) will have fewer variables (variance).

### 2.8. Pretrained Models

One of the significant problems in the field of medical research is the lack of data. But this problem can be overcome using transfer learning. The transfer learning technique minimizes the need for a large dataset by transferring the knowledge from a pretrained model to a new model [32]. The pretrain model consists of trainable and nontrainable layers. While training the pretrained model using a new dataset, the trainable initial layers are replaced by the new layer.

It is necessary to verify the history of the training session in order to test the model. For this TensorFlow, the plot_metrics (history) function was used. The values of training loss, training accuracy, training F1 score, validation loss, validation accuracy, and validation F1 score are provided by the function history.keys().

The accuracy classifier is evaluated with an accuracy metric. The total amount of data that provides accuracy is divided by the amount of correctly classified data. Different values, such as True Positive (TP), False Positive (FP), True Negative (TN), and False Negative (FN), have been used to estimate the accuracy of this study.

(2) $$\begin{array}{c} \text{Accuracy}=\frac{TP+TN}{TP+\;TN+\;FP+FN}. \end{array}$$

In a nutshell, validation and training accuracy indicate how well the model performed during the training and validation phases. The loss function depends on the formula that was followed to calculate the loss in the training or validation phase. The few common ways to calculate loss are binary cross-entropy, squared error loss, and absolute error loss. In the proposed method, the binary cross-entropy method was employed. The negative average of the log of the correct predicted probability is called binary cross-entropy (Figure 6).

(3) $$\begin{array}{c} \text{logloss}=-\frac{1}{N}\sum_{i}^{N}\sum_{j}^{M}yij\text{ log}\left(pij\right). \end{array}$$

Here, N is the number of rows and *M* is the number of classes.

An F1 score is used to measure the accuracy of a model on a dataset. It is determined by the calculated mean of recall and precision.

(4) $$\begin{array}{c} F1-\text{score}=2\times \frac{\text{recall}\times \text{precision}}{\text{recall}+\text{precision}}. \end{array}$$

### 2.9. Explainable AI

In the healthcare area, the ethical issue of AI transparency and a lack of trust in AI systems' black-box functioning demand the use of explainable AI models. XAI methods are AI methods that are used to explain AI models and their predictions [33].

Explainable AI is one of the preeminent prerequisites for implementing responsible AI, a methodology for deploying AI approaches in real life while maintaining model explainability and responsibility. Ethical standards [34] must be embedded in AI applications and processes to use AI responsibly, and AI systems must be built on trust and transparency.

Two research areas are particularly active in addressing this problem: the XAI field and the visual analytics community. Conversely, visual analytics solutions are designed to assist users in understanding and interacting with ML models by offering visualizations and tools that make exploring, analyzing, interacting with, and comprehending ML models easier. As a result, collaboration between the visual analytics and XAI communities is becoming increasingly vital.

Because LIME is model-agnostic, it can be used for various DL models [35]. LIME approximates the model's local linear behavior, which implies it can explain any CNN or natural language processing (NLP) model. Choosing a model-agnostic explainable AI algorithm was critical because the proposed method went through several comparisons between different DL methods. To export the result of a model, the LIME algorithm employs submodular selection. The approach accepts two variables and first explains the weights of responsible features using a sparse linear explanation. Second, the significance of these traits is calculated directly and then optimized using greedy algorithms. The argmax function returns the final feature weight.

## 3. Results and Analysis

After completing the data augmentation process, the models are trained using the Kaggle platform. The Kaggle kernel consists of an Nvidia P100 GPU, with 16 gigabytes of GPU memory and 12 gigabytes of RAM. Each model has been trained with 35 epochs for each fold while training using the cross-validation technique. Adam is implemented as an optimizer, and binary cross entropy is employed for model training as a loss function.

As the dataset has an imbalanced class distribution, every model is trained using stratified k-fold cross-validation. The whole dataset is split three-fold, and the 2nd fold performance matrix score is taken for each model. The score is given in Table 1.

After observing Table 1, it can be stated that InceptionResNetV2 achieved a training accuracy of 99.14%, which is the highest training accuracy compared to other trained models, and a validation accuracy of 95.64%. ResNet101V2 and InceptionV3 also performed well. InceptionV3 achieved a training accuracy of 98.38% and a validation accuracy of 96.65%, the highest validation accuracy compared to other trained models. ResNet101V2 achieved a training accuracy of 98.61% and a validation accuracy of 95.89%. VGG-19 achieved a training accuracy of 96.14% and a validation accuracy of 94.88%, the lowest among all trained models.

InceptionResNetV2 achieved a train loss of 2.78%, the lowest of other trained models. InceptionV3 achieved a train loss of 4.33%. However, InceptionV3 achieved a lower validation loss than InceptionResNetV2. InceptionV3 had a validation loss of 10.48%, while InceptionResNetV2 had a validation loss of 16.42%. ResNet101V2 achieved a train loss of 3.33% and a validation loss of 15.59%. VGG-19 achieved a train loss of 10.60%, the highest compared to other trained models, and a validation loss of 14.25%, lower than ResNet101V2.

In medical image classification, test set accuracy is important as test set accuracy is evaluated by the performance in the unknown dataset. According to Table 2, InceptionV3 achieved the highest test set accuracy. InceptionResNetV2 achieved a test set accuracy of 80.02%. All the models performed well since all the hyperparameters, batch size, and epoch size were kept exactly the same for better comparison between the models. It comes down to model architecture and model complexity. Resnet101V2 achieved 78.26% test set accuracy as it is of medium complexity, but VGG19 scored slightly lower with 77.88% test set accuracy as it is more complex with many layers.

The entire dataset is divided into three folds since every model uses stratified k-fold cross-validation. Hence, the model is trained for three iterations. The plot_metrics() function generates graphs per iteration of each model's training accuracy, loss, and F1 score.

While training using ResNet101V2, the training accuracy has increased rapidly after each epoch. According to the accuracy and loss graph of ResNet101V2 shown in Figure 7, the training accuracy was 50.00% in the first epoch and then increased with each epoch. After 20 epochs, the training accuracy is 95.52%. The model's validation accuracy was 43.56% in the first epoch, and it continued to increase until the last epoch, when it achieved 95.89% in epoch 35. The model loss graph shows that both the training and validation loss lines have gradually decreased. The training loss was 74.99% after the first epoch and 3.33% after 35 epochs.

While training using VGG19, the training accuracy has increased rapidly after each epoch. According to the accuracy and loss graph of VGG19 shown in Figure 8, the training accuracy was 64.63% in the first epoch, then increased with each epoch. After 20 epochs, train accuracy is 91.98%. The model's validation accuracy was 68.20% in the first epoch, and it continued to increase until the last epoch, when it achieved 94.88% in epoch 35. The model loss graph shows that both the training and validation loss lines have gradually decreased. The training loss was 76.66% after the first epoch and 10.60% after 35 epochs.

While training using InceptionResNetV2, the training accuracy has increased rapidly after each epoch. According to the accuracy and loss graph of InceptionResNetV2 shown in Figure 9, the training accuracy was 35.40% in the first epoch and then increased with each epoch. After 20 epochs, train accuracy is 97.47%. The model's validation accuracy was 35.42% in the first epoch, and it continued to increase until the last epoch, when it achieved 95.64% in epoch 35. The model loss graph shows that both the training and validation loss lines have gradually decreased. The training loss was 74.44% after the first epoch and 2.78% after 35 epochs.

While training using InceptionV3, the training accuracy has increased rapidly after each epoch. According to the accuracy and loss graph of InceptionV3 shown in Figure 10, the training accuracy was 39.06% in the first epoch and then increased with each epoch. After 20 epochs, the train's accuracy is 98.82%. The model's validation accuracy was 35.23% in the first epoch, and it continued to increase until the last epoch, when it achieved 96.65% in epoch 35. The model loss graph shows that both the training and validation loss lines have gradually decreased. The training loss was 72.79% after the first epoch and 4.33% after 35 epochs.

Among all the models, InceptionV3 gave the most precise black-box explanation. That is why the InceptionV3 model was picked to identify leukemia cells. The “ImageNet” weight was preferred for the pretrained model weight as it has the most robust training. InceptionV3 takes average pooling and flattens the array. Finally, softmax from the dense layer sample images predicted it as a normal cell or a leukemia blast cell. In the proposed method, LIME is applied, and visual interpretation is used for describing the model. LIME is a model-agnostic algorithm that approximates the local linear behavior of the model, which means it can explain any model of CNN and NLP. An explanation has to be presented so that a human being can easily understand it.

Figure 11 is a sample taken to predict and later explain with the LIME algorithm. The model predicted that this sample image would be ALL. The proposed model takes the highest value as a classification result for prediction. In the case of this sample, the maximum value was 0.99 for ALL. So, the prediction was an ALL image.

A segmentation method was employed to divide the example image into separate sections to see if the model could accurately read it. It also tells us what the sample image represents to the model. By observing the segmentation result, one can easily tell the separation between the foreground and background of the sample image.  Figure 12 shows the sample cell is in the middle with a circular shape highlighted in red.

After that, the 3D image boundary needed to be verified to understand the model's reliability. A scikit-learn image segmentation function was carried out for the 3D boundary. This returns the sample image with its boundaries highlighted between labeled regions. In Figure 13, the boundary is clearly labeled around the sample image to create a 3D depth around the cell. This represents the model's awareness that the intended target is correct.

The LIME algorithm is model-agnostic and can explain both classification and regression models. The proposed model uses the LIME image explainer. The image has to be a 3D NumPy array for this package to work. It explains image prediction by sampling from 0 and then inverting the mean-centering and scaling operations. As the proposed model solves a classification problem, it samples the training distribution, and when the value is the same, it makes a binary feature that is 1. After the explainer is set, the instance from lime_image generates neighborhood data. After learning the weight of the linear models locally, explanations can be extracted from the model. Top_labels show the highest weight of the prediction probability considered for that particular sample image. Finally, the model can explain the major weight behind any prediction. For the above sample image, the model puts more weight on that which is highlighted in red, as shown in Figure 14.

By highlighting this, any doctor can verify if the model was right in predicting all of the sample images. Also, in Figure 15, only the weighted part is more prominent by isolation. This makes the image's explanation more understandable.

The accuracy of the proposed model (InceptionV3) was 98.38%, and the F1 score was 98.39%. The training loss in the final epoch for the model was 4.33%, and the validation loss was 10.48%, with the most explicit Black Box explanation. Moreover, InceptionV3 achieved the highest validation accuracy and F1 score with the lowest validation loss compared to all other trained models.

The best-trained models used in this paper were compared to those mentioned above. The accuracy is given in Table 3. With the help of XAI, the accuracy of all the trained models is sufficient to diagnose leukemia with ease.

The paper used the DCNN method [7], but the accuracy graph was inconsistent, resulting in quite a few large model losses. The proposed model's accuracy graph is consistent. Again, the research [8] applied different DCNN models but did not mention any loss function. The submitted model has a shallow model loss. The study [12] has a model accuracy of 88.69% using histopathological transfer learning, and the study paper [13] had a batch size of 10, which is much lower than usual with only 6 epochs. The mode discussed here has a larger batch size and is trained with more iterations. Research material [15] was applied to a vision transformer, but the proposed model was evaluated with explainable AI, which is more reliable. The groundwork [16] chose the BigDL method, but any evaluation matrix was missing. The proposed method has more contributing factors to a reliable and effective model in these cases.

On account of train accuracy, InceptionV3 has the second-highest score but has the highest validation accuracy and validation F1 score. Furthermore, the InceptionV3 model provided the best fit for XAI, which is more important in medical fields. That is why, for the described method, InceptionV3 was preferred above the rest of the compared models.

## 4. Conclusion

This paper proposed a novel and efficient system, a diagnostic approach for ALL, that compares different transfer learning models to identify malignant and normal cells to assist doctors in diagnosing ALL. The proposed system provides 98.38% accuracy in diagnosing ALL in patients. The result indicates that the model provided more accurate results. By comparing different transfer learning models, they had a more balanced classification capacity that could kick start using different transfer learning models to diagnose ALL. This method also uses LIME to describe which component of the image from the dataset caused the model to produce specific classifications, ensuring the model's validity and reliability. Therefore, the proposed approach gives clinicians a reliable way to diagnose whether or not a patient has leukemia. This system can be used to make an initial ALL diagnosis, after which further testing can be done. The method proposed in this study is a highly promising methodology to identify ALL. In the future, multimodeling and model stacking can be used to develop the model further. With the introduction of newer deep learning models, advanced work will dramatically improve the overall state of this system and its explanation. Also, increasing the size of the dataset and balancing the number of data cells can improve the accuracy. It will provide behavioral inferences and useful insights into deep network operations. This will build trust in DL systems as well as allow for system behavior understanding and improvement.

## Figures and Tables

**Figure 1:** (a) Normal cell. (b) Leukemia blast cell.

**Figure 2:** Block diagram of the proposed method.

**Figure 3:** Augmented sample images.

**Figure 4:** Architecture of InceptionV3.

**Figure 5:** Difference between traditional machine learning and transfer learning.

**Figure 6:** System architecture.

**Figure 7:** Accuracy (a), loss (b), and F1 score (c) of ResNet101V2.

**Figure 8:** Accuracy (a), loss (b), and F1 score (c) of VGG19.

**Figure 9:** Accuracy (a), loss (b), and F1 score (c) of Inception ResnetV2.

**Figure 10:** Accuracy (a), loss (b), and F1 score (c) of InceptionV3.

**Figure 11:** Sample cell.

**Figure 12:** Model segmentation.

**Figure 13:** Model boundaries.

**Figure 14:** Image temperature.

**Figure 15:** Image temperature (positive only).

**Table 1:** Model accuracy, loss, and F1 score.

Model	Accuracy	Loss	Validation accuracy	Validation loss	F1 score	Validation F1 score
ResNet101V2	0.9861	0.0333	0.9589	0.1559	0.9861	0.9588
VGG19	0.9614	0.1060	0.9488	0.1425	0.9615	0.9487
InceptionResNetV2	0.9914	0.0278	0.9564	0.1642	0.9914	0.9563
InceptionV3	0.9838	0.0433	0.9665	0.1048	0.9839	0.9665

**Table 2:** Test set accuracy and F1 score.

Model	Test set accuracy	Test set F1 score
ResNet101V2	0.7826	0.7770
VGG19	0.7788	0.7695
InceptionResNetV2	0.8002	0.7980
InceptionV3	0.7981	0.7955

**Table 3:** Result comparison with previous work.

Paper	Accuracy (%)	This paper's accuracy (%)
In paper [7]	80.40	98.38
In paper [8]	96.58	
In paper [12]	88.69	
In paper [13]	96.15	
In paper [15]	99.03	
In paper [16]	96.42	

## Data Availability

The data used to assist the finding of this study are openly accessible at https://www.kaggle.com/andrewmvd/leukemia-classification.
